# The Distribution and Composition of Colonoscopy Providers in Australia

**DOI:** 10.7759/cureus.22104

**Published:** 2022-02-10

**Authors:** Moon Soo Choi, Michael A van der Mark, Kevin Hung

**Affiliations:** 1 General Surgery, Bundaberg Base Hospital, Bundaberg, AUS

**Keywords:** colonoscopy, general surgery, gastroenterology, rural health

## Abstract

Introduction: Colorectal cancer is a common cause of cancer in Australia. Also, patients living in regional and rural areas are diagnosed later and have poorer outcomes compared to their metropolitan counterparts. The purpose of this study is to determine the distribution of the workforce providing colonoscopies for the Australian population.

Methods: A cross-sectional observational study of the medical practitioners certified by the conjoint committee for the recognition of training in gastrointestinal endoscopy (CCRTGE) was performed. Data regarding their specialty and principal place of practice was collected. The principal place of practice was stratified with the Modified Monash Model (MMM) of rurality and the local government association’s classifications of rural and urban areas.

Results: As of March 2021, there were 2698 medical practitioners listed as being recognised in the field of adult colonoscopies by the CCRTGE. Of these, 2123 were found to still have active specialist registration with the Australian Health Practitioner Regulation Agency (AHPRA). In the capital city Local Government Areas (LGAs), there was an endoscopist every 0.33 km^2^ to 62.05 km^2^. In the rural LGAs, there was an endoscopist every 23,382 km^2^ to 267,780 km^2^. In metropolitan areas, the most common specialty of the endoscopist was gastroenterology whereas in regional cities and remote towns it was general surgery. In very remote towns, general practitioners provided colonoscopy services.

## Introduction

Colorectal cancer is Australia’s third most diagnosed cancer with 17,004 new cases in 2018. It is also the second most common cause of cancer death with 4129 deaths [1]. Colonoscopic removal of polyps in patients with positive screening tests, symptoms of colorectal cancer, and strong family history is an effective way of preventing colorectal cancer or detecting it in its early, surgically curable stages [2]. Effective and cost-efficient screening measures have been put into place internationally including Australia although low participation rates are preventing its full potential [3].

The Australian National Bowel Cancer Screening Program (NBCSP) was started by the Australian Federal Government in 2006 with the aim of prevention and early detection of colorectal cancer. All Australians between the ages of 50 and 74 years are invited to participate in two-yearly immunochemical faecal occult blood testing (iFOBT). If found to be positive, the patient is offered a colonoscopy to remove any polyps prior to becoming cancerous or to facilitate early detection of cancer. Colonoscopies are subsidised by the Australian government’s universal health care insurance scheme “Medicare” and take place in public and private hospitals [4].

Colonoscopies in Australia are provided mainly by medical practitioners though there are a small number of nurse-endoscopists in select pilot hospitals. The Royal Australasian College of Surgeons (RACS), Royal Australasian College of Physicians (RACP), and the Gastroenterological Society of Australia (GESA) created the Conjoint Committee for the Recognition of Training in Gastrointestinal Endoscopy (CCRTGE) in 1990 to provide uniform training and assessment of endoscopy training.

Assessment for recognition of training in colonoscopy involves a logbook of a minimum of 200 lower GI endoscopies consisting of at least 100 complete colonoscopies to the caecum and successful polypectomies in at least 50 patients. This must be completed over a maximum of a five-year period and candidates must gain specialist registration as a surgeon, physician, or general practitioner [5].

Regional and rural Australians have a well-documented disparity of health outcomes with a poorer life expectancy and lower access to general practitioners and medical specialists [6]. In terms of colorectal cancer, regional and rural Australians are found to present in later stages of colorectal cancer and have poorer five-year survival rates when compared to their metropolitan counterparts [7].

Geographic remoteness is defined by the Australian Government Department of Health by the Modified Monash Model (MMM) 2019. The model has seven categories from MM1 (metropolitan areas) to MM7 (very remote areas). This is based on the size of the town and the distance to the nearest large population centre (See Appendix) [8].

Local Government Areas (LGAs) are the third tier of government in Australia under the federal and state or territory governments chiefly responsible for local infrastructure. These LGAs are composed of Local Health Districts (LHDs), which in turn provide health services such as colonoscopies to a local population. There can be some non-concordance with LGAs and LHDs in states like New South Wales though in most states they do align [9,10]. The LGAs can also be divided into state capital city LGAs, urban LGAs, and rural LGAs [11].

In this study, we studied the composition of specialist medical practitioners providing colonoscopies to patients in Australia and their distribution around metropolitan and regional Australia, both in terms of the MMM and their LGA.

## Materials and methods

The list of medical practitioners’ names certified by the CCRTGE to perform colonoscopies was individually searched on the Australian Health Practitioner Regulation Agency (AHPRA) register. The search parameters were medical practitioners with active specialist registration in the field of surgery, medicine, or general practice practising within Australia. When there were two or more practitioners with the same name, it was assumed that the general surgeon or gastroenterologist was most likely to be the practitioner. If there were multiple surgeons or gastroenterologists with the same name, the practitioner was removed. Data regarding their specialty field, postcode and principal place of practice were gathered.

This project has been reviewed by the Research Ethics and Integrity Committee of the University of Queensland and is deemed to be exempt from ethics review under the National Statement on Ethical Conduct in Human Research and relevant University of Queensland policy (PPL 4.20.07).

## Results

The CCRTGE had 2689 practitioners recognised for adult colonoscopies as of March 5, 2021. Practitioners named “Delete Me”, presumably for administration purposes, were removed. Of these, 2290 were found to have specialist registration on AHPRA. Of these, 104 were registered as “non-practising,” “teaching and/or assessing” or re-registered short-term under the coronavirus pandemic response sub-register and were also removed. Of the remaining 2186, 2130 were practising within Australia. Seven practitioners had the same name as other surgeons or gastroenterologists making them indistinguishable and were removed.

Data regarding the remaining 2123 practitioners' specialty field, postcode, and suburb of principal place of practice was gathered. The MMM category and the LGA of each practitioner were attributed. This process is illustrated in Figure 1.

**Figure 1:** Flowchart for Selection of Practitioners Recognised to Perform Colonoscopies

Each specialist group was divided by their respective MMM category (Table 1). In MM1 (metropolitan) areas, the most common type of medical practitioner was a gastroenterologist. In MM2 (regional) to MM6 (remote community), the most common type of practitioner were general surgeons. In MM7, only general practitioners performed colonoscopies.

**Table 1:** Number of Specialists Accredited to Perform Colonoscopies Residing in Each Modified Monash Model Category Note: (a) If dual trained in gastroenterology and another medical specialty, the doctor is considered a gastroenterologist (b) Surgery contains three paediatric surgeons accredited to perform adult colonoscopy, all in Modified Monash Model category 1

	Modified Monash Model Category													
	1		2		3		4		5		6		7	
	N	%	N	%	N	%	N	%	N	%	N	%	N	%
Gastroenterologist	852	50.24	22	12.43	23	14.94	2	5.41	1	4.00	1	12.50	0	0.00
Surgeon	813	47.94	141	79.66	122	79.22	20	54.05	16	64.00	6	75.00	0	0.00
Other Physician	26	1.53	12	6.78	7	4.55	3	8.11	1	4.00	1	12.50	0	0.00
General Practitioner	5	0.29	2	1.13	2	1.30	12	32.43	7	28.00	0	0.00	1	100.00
Total	1696	80.84	177	8.44	154	7.34	37	1.76	25	1.19	8	0.38	1	0.05

As a percentage of endoscopists per MMM category, general surgeons made up the bulk of the colonoscopy workforce in MM2 to MM6 areas (Figure 2). General practitioner endoscopists, while few numerically, provided services mainly to MM5 (medium rural town) and MM6 (small rural town) areas.

**Figure 2:** Graph of Specialty Make-up of Endoscopists Residing in Each Modified Monash Model Category GP: General Practitioner

The endoscopists were divided into their respective LGAs and compared to the population (Table 2). The difference between metropolitan and rural Australia becomes stark. In capital city LGAs, the number of endoscopists ranged from 0.94 to 19.83 per 10,000 population while in rural LGAs, the number ranged from 0 to 0.21 per 10,000 population.

**Table 2:** Population and Endoscopists of the Capital City, Urban, and Rural LGAs of Each State and Territory^ ^Population of people residing in local government areas in 2016-2017, excluding population in unincoporated areas *Australian Capital Territory has no municipalities LGA: Local Government Area

		States and Territories							
		New South Wales	Victoria	Queensland	Western Australia	South Australia	Tasmania	Northern Territory	Australia Capital Territory*
Capital City LGA	Population	205339	128980	1162186	21092	22690	50714	82816	406403
	Endoscopists	53	88	163	22	45	12	17	38
	Endoscopist per 10000	2.58	6.82	1.40	10.43	19.83	2.37	2.05	0.94
Urban LGA	Population	6899621	5507871	3418398	2254804	1439358	310445	73656	
	Endoscopists	646	469	274	148	105	15	2	
	Endoscopist per 10000	0.94	0.85	0.80	0.66	0.73	0.48	0.27	
Rural LGA	Population	502467	300611	194304	314363	223666	155427	80780	
	Endoscopists	9	5	4	3	4	2	0	
	Endoscopist per 10000	0.18	0.17	0.21	0.10	0.18	0.13	0.00	

The concentration of endoscopists in an area (Table 3) also varies greatly depending on the urban and rural nature of each state’s LGAs. In the capital city LGAs, there was an endoscopist every 0.33 km^2^ to 62.05 km^2^ while in rural LGAs this area ranged from 23,382 km^2^ to 267,780 km^2^ excluding the rural Northern Territory, which had an area totalling 1,320,876 km^2^ with no endoscopists.

**Table 3:** Area and Endoscopists of the Capital City, Urban, and Rural LGAs of Each State and Territory^ ^Area does not included unincorporated areas in New South Wales, Victoria, Western Australia, South Australia, Northern Territory *Australian Capital Territory has no municipalities LGA: Local Government Area

		States and Territories							
		New South Wales	Victoria	Queensland	Western Australia	South Australia	Tasmania	Northern Territory	Australia Capital Territory*
Capital City LGA	Area (km^2^)	27	37	1338	9	15	78	142	2358
	Endoscopists	53	88	163	22	45	12	17	38
	Km^2^ per Endoscopist	0.51	0.42	8.21	0.41	0.33	6.50	8.35	62.05
Urban LGA	Area (km^2^)	139807	110263	361401	134058	10410	5141	73656	
	Endoscopists	646	469	274	148	105	15	2	
	Km^2^ per Endoscopist	216.42	235.10	1318.98	905.80	99.14	342.73	36828.00	
Rural LGA	Area (km^2^)	563063	116914	1367206	803340	145222	62693	1320876	
	Endoscopists	9	5	4	3	4	2	0	
	Km^2^ per Endoscopist	62562.56	23382.80	341801.50	267780.00	36305.50	31346.50	-	

## Discussion

We have analysed the specialist makeup and location of practice of Australia’s endoscopists to understand the distribution and density of the nation’s colonoscopy-performing workforce. There is a shortage of healthcare practitioners in Australia with many concentrated in metropolitan or urbanised areas despite rural areas having a greater need for their services.

In the capital city of South Australia, Adelaide, there were 45 endoscopists for a population of 22,690 - an endoscopist for approximately every 500 people. In rural LGAs of South Australia, there were four endoscopists for a population of 223,666 - an endoscopist for approximately 55,000 people. In capital city LGAs such as Sydney City in New South Wales, there is an endoscopist every 0.5 km^2^ while in rural Queensland LGAs with a combined area of 341,801 km^2^, approximately the size of Germany, there are four endoscopists - three of whom are general practitioners and a general surgeon.

It should be noted that the size and population of an LGA are not uniform among states, with some being amalgamations of many abolished local governments. For example, the City of Brisbane is the capital city LGA of the state of Queensland with a population greater than a million. Meanwhile, the City of Sydney, the capital city LGA of New South Wales, only contains approximately 200,000 people despite Sydney as a metropolitan area is far bigger than Brisbane.

Gastroenterologists were mostly found in metropolitan, regional, and large rural towns (MM1-MM3) while surgeons were distributed into metropolitan to small rural towns (MM1-MM6). General practitioners accredited to perform colonoscopies were few in number. However, they made up a significant portion of the endoscopy workforce in MM4 (medium rural towns) to MM7 (very remote communities). Nurse-endoscopists are a novel program in which non-physician health professionals are credentialled to perform colonoscopies under the supervision of gastroenterologists. However, in Australia, these programs are situated in metropolitan areas and are unlikely to make a significant contribution to regional and rural colonoscopy figures [12].

There are significant limitations to this study. Chiefly, the distribution of endoscopists does not give any idea of their individual level of activity as the practitioner may not perform many colonoscopies or perform any for the NBCSP. This study solely looked at the physical distribution of practitioners, not the services provided. The register with the CCRTGE is voluntary and the exact number of practitioners electing to stay off the register is not made public. However, this number was not thought to be large as many employers utilise this list for employment purposes.

Another aspect not considered in this analysis is that endoscopists may not work solely at their principal place of practice or may perform outreach services in rural and regional areas as part of their employment. Gastroenterology outreach programs provide specialist gastroenterology services including endoscopy to rural health services and the specialists involved would not have their regional and rural activities reflected in this study [13]. Also, metropolitan LGAs serve as referral centres for smaller regional centres.

Lastly, the CCRTGE is currently undergoing a re-accreditation process with all endoscopists required to perform 150 colonoscopies in three years with evidence of sufficient caecal intubation and polypectomy rates to maintain their recognition of training. This may find endoscopists without a sufficient caseload lose their accreditation in the future [14].

This study suggests that the disparity of Australia’s colorectal cancer outcomes between metropolitan and rural populations may be in part due to the difficulty of accessing medical practitioners trained in colonoscopy. Comparing the rate of NBCSP participation and colorectal cancer outcomes of non-metropolitan areas with and without an endoscopist is an idea for further research.

## Conclusions

We have studied the specialty composition and distribution of medical practitioners trained to perform colonoscopies in Australia. There was a significant shortage of endoscopists in regional and remote areas. General practitioners credentialled in colonoscopies provide this valuable service in very remote communities. Regional cities and rural towns are largely serviced by general surgeons. A proportionately larger number of endoscopists in metropolitan centres are gastroenterologists. This study may provide a foundation for further studies characterizing the national endoscopist workforce and work addressing healthcare inequities in rural Australia. 

## Appendices

**Table 4:** Modified Monash Model 2019 ASGS-RA: Australian Statistical Geography Standard-Remoteness Area; MM: Modified Monash Source: Australian Government Department of Health [8]

Modified Monash category	Inclusions
MM 1	All areas categorised ASGS-RA1.
MM 2	Areas categorised ASGS-RA 2 and ASGS-RA 3 that are in, or within 20km road distance, of a town with a population greater than 50,000.
MM 3	Areas categorised ASGS-RA 2 and ASGS-RA 3 that are not in MM 2 and are in, or within 15km road distance, of a town with a population between 15,000 and 50,000.
MM 4	Areas categorised ASGS-RA 2 and ASGS-RA 3 that are not in MM 2 or MM 3 and are in, or within 10km road distance, of a town with a population between 5,000 and 15,000.
MM 5	All other areas in ASGS-RA 2 and 3.
MM 6	All areas categorised ASGS-RA 4 that are not on a populated island that is separated from the mainland in the ABS geography and is more than 5km offshore. Islands that have an MM 5 classification with a population of less than 1,000 (2019 Modified Monash Model classification only).
MM 7	All other areas; that being ASGS-RA 5 and areas on a populated island that is separated from the mainland in the ABS geography and is more than 5km offshore.
